The article "Effect of Carbon Dioxide on Bispectral Index of EEG under Intravenous Target-Controlled Anesthesia Based on Intelligent Medical Treatment" was retracted in 2023. Reasons: signs of a paper mill; suspected computer-generated content; unreliable results or conclusions; lack of ethics approval or compliance.

# Effect of Carbon Dioxide on Bispectral Index of EEG under Intravenous Target-Controlled Anesthesia Based on Intelligent Medical Treatment

**DOI:** 10.1155/2022/4696128

**Published:** 2022-03-27

**Authors:** Aizhi Li, Qunhui He, Rulin Li, Yu Chen, Weiwei Xu

**Affiliations:** ^1^Yantai Yuhuangding Hospital, Anesthesiology Department, 264000 Shan Dong, China; ^2^Yantai Zhifu Hospital, Anesthesiology Department, 264000 Shan Dong, China

## Abstract

Laparoscopic surgery has the advantages of less trauma and quick recovery, and it is more and more favored by surgeons and patients in clinical practice. However, the impact of carbon dioxide pneumoperitoneum on the body during laparoscopic surgery has attracted the attention of many scholars. Pneumoperitoneum can cause increased cerebral blood flow and increased intracranial pressure, cerebral metabolic rate is highly correlated with blood carbon dioxide partial pressure, and cerebral metabolism without cardiopulmonary bypass is linearly correlated with the depth of anesthesia. Electroencephalographic (EEG) bispectral index (BIS) is a signal analysis method, which can directly measure the effect of drugs on the cerebral cortex and reflect the depth of anesthesia. Based on this, this study takes smart medical treatment as the background and uses the improved BP neural network as a tool to explore the effect of carbon dioxide on EEG bispectral index under intravenous target-controlled anesthesia. The main purpose is to observe the correlation between arterial blood carbon dioxide partial pressure and EEG bispectral index under propofol target-controlled anesthesia during retroperitoneal laparoscopic surgery. The experimental results show that the model proposed in this study can efficiently and accurately obtain the size of the influencing factors, which provides a clinical basis for the anesthesia management and anesthesia depth regulation of carbon dioxide pneumoperitoneum laparoscopic surgery.

## 1. Introduction

Anesthesia depth assessment is always an important issue with the development of anesthesiology. It is directly related to the safety of patients during operation and postoperative outcome [1]. There are many methods to monitor the depth of general anesthesia. However, there is no method that can directly, accurately, and dynamically reflect the depth of anesthesia. In the past, the depth of anesthesia was indirectly reflected by monitoring the changes in hemodynamics. It was also useful to use primitive electroencephalogram (EEG), auditory evoked potential, electromyography, changes in esophageal contractility, pupillary reflex, comprehensive analysis of various variations, and multifactor logic equation analysis of microcomputer. However, there has been no direct method to determine the effect of anesthetics on the central nervous system. Taking the clinical use of muscle relaxants as the boundary, its development can be divided into two stages: in the former stage, anesthetists evaluate the depth of anesthesia by observing the changes in patients' autonomic nervous system (heart rate, blood pressure, tears, pupil size, etc.) and somatic reaction during anesthesia [2]. It is often necessary to meet the muscle relaxant effect required by surgery at the cost of deepening anesthesia. Therefore, there is a risk of too deep anesthesia; in the latter stage, the use of muscle relaxants may mask some clinical signs (such as body movement reaction) of patients during anesthesia, so that some “inadequate anesthesia” cannot be found in time, resulting in intraoperative awareness, which will cause physical and mental damage to patients [3].

So far, the purpose and content of anesthesia depth monitoring include preventing potentially dangerous hemodynamic changes, preventing intraoperative body movement, eliminating intraoperative awareness, and regulating the number of anesthetic drugs [4]. In recent years, the focus of anesthesia depth monitoring has turned to electroencephalogram (EEG) analysis. Conventional EEG can reflect the activity of the cerebral cortex and subcortical nervous system, but the operation is complicated, susceptible to external interference, difficult to analyze data, and difficult to routinely apply to Clinical determination of anesthetic effects [5]. In recent years, with the application of microcomputers and the development of EEG analysis technology, the application of EEG technology in clinical anesthesiology has received attention again, and different EEG parameters such as bi-frequency index have been derived, which can reflect the brain more accurately and timely [6]. Among them, the electric bispectral index (BIS), which has been widely studied, is known as a useful index to reflect the depth of anesthesia, and it has its own characteristics in clinical applications [7]. A large number of studies have shown that the bispectral index (BIS) is currently a very reliable indicator for evaluating the depth of sedation in anesthesia. BIS has received much attention and research in the field of clinical anesthesia [8]. This article intends to evaluate its application in anesthesia depth monitoring.

At present, the research on carbon dioxide (CO_2_) pneumoperitoneum mostly focuses on the impact on physiology, and few people pay attention to the impact of CO_2_ pneumoperitoneum on the depth of anesthesia. This research study is conducted to explore whether CO_2_ pneumoperitoneum has a synergistic or antagonistic effect on the depth of anesthesia and draw a statistically significant difference, which is an exploration in a new direction.

## 2. Related Work

### 2.1. Research Status of Monitoring Mechanism

There are two forms of electrical activity, spontaneous EEG activity and induced EEG activity. The main differences between the two are as follows: (1) spontaneous EEG is the EEG activity in a quiet state without any external stimulation, which often shows continuous rhythmic potential changes; evoked EEG is a relatively limited potential change generated in a certain area of the skin layer under external stimuli such as sound, light, and electricity. (2) The amplitude of spontaneous EEG is high, 50–100 Hz, no signal stimulation is required, and the waveform is continuous, so there is no time-phase relationship [9]. The recording adopts direct amplification, and its waveform has only physiological significance; the evoked EEG intensity is weak, only 0.3∼20 V, and there must be signal stimulation. The waveform is limited and has a time-locked relationship with the stimulation. The recording adopts synchronous superposition, and its waveform has not only physiological significance but also specific anatomical positioning and psychological significance. BIS belongs to spontaneous EEG monitoring [10].

The shape of brain wave shows the spontaneous and rhythmic electrical activity of brain cell group, which is generally described by the characteristics of amplitude, frequency, and phase. During general anesthesia, EEG frequency changes sequentially with the deepening or shallowing of anesthesia and has a functional relationship with anesthetic concentration, so it can be used to reflect the depth of anesthesia [11]. However, in the early stage, the time-domain characteristics of EEG were mostly used to reflect the depth of anesthesia, mainly analyzing the geometric properties of EEG waveform. With the maturity of fast Fourier transform technology, more and more EEG frequency domain features can be used to reflect the depth of anesthesia, convert the original EEG signal with time-to-amplitude relationship into frequency-to-power relationship, and derive multiple digital quantization parameters, such as dual frequency index (BIS), edge frequency (SEF), and intermediate frequency (MF). The phase-locking energy is subtracted from energy and expressed as the ratio of double-wave spectral density in 0∼30 Hz band. Finally, a quantitative index is obtained [12]. On the one hand, the EEG characteristics of PBIS are reflected in the amplitude and frequency characteristics, and on the other hand, they are reflected in the waveform and phase characteristics. Accordingly, EEG analysis methods are also divided into frequency-domain analysis and time threshold analysis [13]. The traditional processing method is to use fast Fourier transform (FFT) to convert the change in EEG amplitude into the change in EEG power, that is, spectrum analysis. However, FFT is a typical linear analysis method, which is suitable for stable and nonrandom normal distribution signals, while EEG activity is a random skew distribution signal. Therefore, there are some limitations in analyzing EEG with this linear analysis method. BIS is a quantitative analysis index of EEG including frequency, amplitude, and phase [14]. The advantage of its monitoring is to maintain and quantify the nonlinear relationship of the original EEG, so it can better retain the functional information of the original EEG. The observation is simple and easy to use. Bispectral analysis is to quantify the phase coupling between EEG frequencies [15].  Figure 1 shows the schematic diagram of EEG signal and bispectral index.

Including frequency and amplitude information, phase coupling is the characteristic of nonlinear behavior. Therefore, bispectral analysis can accurately control and quantify the linear and nonlinear changes between signals, and it can more accurately reflect the changes in anesthesia depth. The changes in frequency and power of many anesthetics do not form a simple relationship with dose [16]. Low doses of benzodiazepines or propofol usually cause high-frequency activation, showing a net increase in frequency in the power spectrum, while higher doses of thiopental or isoflurane can cause explosive inhibition and a net decrease in power. BIS decreased during natural sleep, but it was impossible to achieve the degree of inhibition caused by high-dose propofol, sodium thiopental, or volatile anesthetics [17]. Many studies have found that with the deepening of anesthesia, the electrophysiological activities of central nerve cells change significantly. Therefore, BIS has an important value in EEG signal analysis. BIS is a dimensionless simple variable, representing fully awake state and completely no EEG activity state, respectively.

### 2.2. Clinical Application

It is found that BIS can better reflect different sedation (sleep) depths. Whether there is awareness, memory, and implicit memory in anesthesia depends on the sedation depth in anesthesia. It is found that the BIS value is 75∼90 in light sleep, 75∼92 in rapid eye movement, and 20∼70 in slow-wave sleep [18]. It is more advantageous to distinguish the existence and disappearance of consciousness. The sedation level depends on the inhibition degree of drugs on the cerebral cortex, which is related to the concentration of sedative and hypnotic drugs in the effective part (brain). BIS has a good correlation with the plasma concentrations of propofol and sevoflurane, which provides a theoretical basis for monitoring the depth of anesthesia (sleep). Because BIS has the above advantages in monitoring the depth of sleep (anesthesia), it helps to reduce blindness and improve safety in clinical anesthesia.  Figure 2 represents the basic EEG monitoring [19].

However, more attention should be paid to the body movement in the anesthesia maintenance stage: on the one hand, due to the complex relationship between anesthesia factors (sedation, analgesia, and muscle relaxation) and surgical stimulation factors, and the existence of individual differences in patients, it is more difficult to manage body movement at this stage [20]. On the other hand, the body movement management at this stage is more necessary: because at this time, the body movement not only affects the surgical operation but also may cause accidents for some fine operations. Unfortunately, there are few studies on this stage [21]. The results of the above studies show that BIS monitoring improves the quality of anesthesia and is convenient for drug control, but BIS evaluation of anesthesia depth obviously depends on the anesthesia method used, mainly reflecting the patient's sedation or sleep depth. Patients with high-dose opioids may still show shallow anesthesia when there is no obvious somatic reaction to skin incision, indicating that BIS is different in evaluating the effects of analgesics and sedatives [22]. In conclusion, BIS changes with the increase or decrease in anesthetic concentration and dose and with the increase or decrease in surgical stimulation intensity.

### 2.3. Research Status of Impact Assessment Algorithm

The machine learning algorithm is an important content in the field of data analysis. We have frequent contact with the machine learning algorithms in our daily work. The machine learning algorithm classification is to subdivide the samples to be detected into the most appropriate class. The following introduces the common machine learning classification algorithms. The decision tree classification algorithm is widely used in our daily life because of its simple implementation principle. The decision tree algorithm uses tree structure for classification and decision-making. The important content of the decision tree algorithm is to improve the accuracy and reduce the scale of the algorithm [23]. The following describes the construction steps of the decision tree, which mainly includes two parts. The first is the generation of the decision tree, which is generally obtained from the training sample set, in which the sample data set has high requirements [24].

The Bayesian classification is a statistical classification method, which involves the knowledge of probability. It mainly achieves the classification effect by successfully classifying a given set of test elements into a specific category [25]. Among them, the most commonly used method in the Bayesian algorithm is the naive Bayesian algorithm. The naive Bayesian method is a classification method that assumes the independence of feature conditions under the condition of the Bayesian algorithm. It is the simplest and most commonly used Bayesian classification algorithm. The advantage of the naive Bayesian algorithm is that it needs less estimated parameters and is not sensitive to missing data; however, its accuracy mainly depends on the assumption of independence between attributes, and the algorithm has no classification rule output [26].

An artificial neural network is an algorithm that imitates the neural structure of the biological brain and its information transmission and processing. It is composed of input and output units organized together, and any connection of each unit has a weight. In the e-learning stage, the one-to-one correspondence among various categories is realized through the continuous adjustment of the weight [27]. BP neural network is the most widely used form of neural network at present. BP neural network is a network trained based on an error back propagation algorithm. Its advantage is that it has a strong nonlinear mapping ability. Secondly, the number of hidden layers and the number of neural units in each layer of the network can be unlimited, but the performance will be different with the different structures. This study focuses on the research of BP neural network algorithm, which will be further elaborated in the following chapters [28].

Apart from the use of AI models in different domains, intelligent models have been proposed for identifying the ways how to reduce CO_2_ in the environment to be safe from its bad impacts on the human health [29]. Similarly, intelligent decision models have been proposed and implemented to realize the scenario of physical activities recommendations and diabetes' type prediction using multimodal hybrid reasoning [30] and roughest reasoning [31], respectively.

## 3. Impact Assessment Model

This section introduces the overall structure of the impact assessment model of optimizing BP neural network based on the improved grey wolf algorithm. Firstly, it introduces the basic principle of grey wolf algorithm, then introduces how to improve grey wolf algorithm, and finally introduces how to optimize BP neural network based on the improved grey wolf algorithm.

### 3.1. Principle of Grey Wolf Algorithm

Grey wolf optimization algorithm is a new swarm intelligence optimization algorithm, which imitates the leadership and hunting mode of grey wolf group in nature. According to the fitness value, GWO algorithm divides wolves into four categories: *α*,  *β*, *δ*, and  *ω*. Among them, *α* is the leader of the grey wolf, responsible for the decision-making of the whole wolf group:  *β* is the second best Grey wolf, follows the orders issued by *α* in the wolf group, and also leads the subordinate wolf group. *δ* is the third grey wolf to help make decisions and is responsible for assisting *α* and *β* wolves to complete the hunting of prey: other grey wolves belong to *ω*, which is the basis of the wolf group and must obey the decision of the leadership. When catching prey, grey wolves  *α*, *β*, and *δ* chase prey directly. The remaining grey wolves follow the first three types of grey wolves to track and surround their prey. In the GWO algorithm, the position of prey corresponds to the solution of the problem. The research shows that the GWO algorithm is obviously superior to particle swarm optimization algorithm, genetic algorithm, and other intelligent optimization algorithms in finding the global optimal solution. The mathematical model of grey wolf optimization algorithm is as follows:

(1) $$\begin{array}{c} D=\left|K\cdot X_{P}\left(t\right)-X\left(t\right)\right|,\\ X\left(t+1\right)=X_{p}\left(t\right)-A\cdot D, \end{array}$$

where *t* represents the current number of iterations. *X*_*P*_ is the location of prey; *X* is the position vector of grey wolves in the wolf pack; and *A* represents the convergence factor. *A* and *K* are calculated as follows:

(2) $$\begin{array}{c} A=2a\cdot d_{1}-a,\\ K=2d_{2}, \end{array}$$

where components of *a* are linearly decreased from 2 to 0 over the course of iterations and  *d*_1_ and *d*_2_  are random vectors in [0, 1]. When the location of the prey is determined, grey wolf *α* leads grey wolves *β* and *δ* to guide the wolves to surround the prey. Since  *α*, *β*, and *δ* are closest to the prey, the approximate position of the prey can be judged from the position of the three wolves. The mathematical expression is as follows:

(3) $$\begin{array}{c} D_{\alpha }=\left|K_{1}\cdot X_{\alpha }\left(t\right)-X\left(t\right)\right|, \end{array}$$

(4) $$\begin{array}{c} D_{\alpha }=\left|K_{2}\cdot X_{\beta }\left(t\right)-X\left(t\right)\right|, \end{array}$$

(5) $$\begin{array}{c} D_{\delta }=\left|K_{3}\cdot X_{\delta }\left(t\right)-X\left(t\right)\right|. \end{array}$$

Among them, *X*_*α*_, *X*_*β*_, and *X*_*δ*_ represent the current positions of grey wolves *α*, *β*, and *δ*, respectively. *K*_1_, *K*_2_, and *K*_3_ are random vector coefficients, and *X* represents the current position vector of grey wolf. The following equation represents the forward distance and direction of other grey wolves *ω* towards grey wolves *α*, *β*, and *δ*, respectively:

(6) $$\begin{array}{c} X_{1}=X_{\alpha }-A_{1}\cdot D_{\alpha }\\ X_{2}=X_{\beta }-A_{2}\cdot D_{\beta }\\ X_{3}=X_{\delta }-A_{3}\cdot D_{\delta }\\ X\left(t+1\right)=\frac{\left(X_{1}+X_{2}+X_{3}\right)}{3}. \end{array}$$

Among them, *X*_1_ refers to the position update of *ω* wolves led by grey wolf *α*, *X*_2_ refers to the position update of *ω* wolves led by grey wolf *β*, and *X*_3_ refers to the position update of *ω* wolves led by grey wolf *β*, and equations (3) and (4) represent the updated grey wolf position, and equation (6) represents the final position of prey. According to the above equation (especially the calculation of forward distance and direction), the grey wolf group gradually approaches the prey and catches the prey. The implementation process of grey wolf algorithm is as follows:

1. Firstly, the grey wolf population is initialized to generate *n* grey wolf positions. Then, *A*, *a,* and *K* are initialized, and the maximum number of iterations *t*_max_ is determined.
2. The fitness value of each Grey wolf individual is calculated, the position of the grey wolf according to equations (4)–(6) is updated, the fitness values of each grey wolf individual is compared, and the optimal solution of the fitness value, the suboptimal solution, and the third optimal solution are found.
3. The values of *A*, *a*, and *K* are updated.
4. Whether the current number of iterations *t* is within the maximum number of iterations is compared. If *t* < *t*_max_, step 2 is processed.
5. Otherwise, process should be ended.

The grey wolf algorithm flow is shown in Figure 3.

Many researchers have proved that grey wolf optimization algorithm is superior to particle swarm optimization algorithm, genetic algorithm, and other intelligent optimization algorithms in forming the global optimal solution of the problem. However, because the grey wolf algorithm itself is easy to fall into local optimization, its convergence accuracy is not high. At present, the grey wolf algorithm belongs to a new swarm intelligence algorithm, which has a good room for improvement in convergence accuracy and efficiency. Therefore, the improvement of grey wolf algorithm plays a very important role in the further research of grey wolf algorithm in the future. The improvement of grey wolf algorithm will be described in detail as follows.

### 3.2. Improved Grey Wolf Algorithm

Grey wolf algorithm is proposed and more and more applied to real life because of its convenient parameter setting, good robustness, and good optimization effect. However, because it is easy to fall into local optimization in the later stage, the accuracy is affected. This disadvantage is not only a problem in grey wolf algorithm, but also a common consistency problem in general swarm intelligence optimization algorithm. The common problem of swarm intelligence optimization algorithm is the disharmony between global and local search performance. This will lead to the reduction in convergence accuracy and performance. A swarm intelligence optimization algorithm with strong generalization ability and wide applicability must have a strong coordination mechanism of global and local search performance.

The control factor *A* in grey wolf algorithm is a very important factor for coordinating the performance of global search and local search. Therefore, this section mainly introduces the optimization of control factor *a*. Therefore, the calculation of control factor needs to be optimized and improved. In this section, a nonlinear control factor algorithm based on logarithmic function is proposed for the control factor of grey wolf algorithm, and its equation is shown as follows:

(7) $$\begin{array}{c} a=\;\log_{2}\left(4-\frac{3t}{t_{\max}}\right), \end{array}$$

where parameter *t* is the number of iterations, and parameter *t*_max_ is the maximum number of iterations. The improved control factor *A* has changed from linear decline to nonlinear decline. The initial control factor *A* is monotonic, and the rate in the decline process is consistent. The improved control factor *a* changes according to the law of logarithmic decline. This can better coordinate the global and local search capabilities and more in line with the change trend and convergence process of control factors in the experiment.

The first three types of wolves in the grey wolf algorithm are *α*, *β*, and *δ*, respectively. During the implementation of the grey wolf algorithm, the three types of wolves *α*, *β*, and *δ* led other wolves to *ω* track prey. In the experiment, the three types of wolves play the same guiding and leading role, regardless of grade. However, in terms of the principle of the grey wolf algorithm itself, the three types of wolves  *α*, *β*, and *δ* should be limited by hierarchical order; that is, wolf  *α*, wolf *β*, and wolf *δ* have different degrees of guidance for other wolves  *ω*. Grey wolf *α* is the leader, and grey wolves *β* and *δ* mainly help wolf *α* make decisions. This leadership role is closely related to the appetite level. In the implementation process of grey wolf algorithm, the corresponding fitness values of *α*, *β*, and *δ* calculated through the fitness function are equivalent to the three optimal solutions of the function, which does not reflect the leadership degree between grey wolves, which also reduces the convergence speed of grey wolf algorithm, and then, it is easy to form a local optimal problem. In view of this, this section realizes the dynamic follow-up of grey wolf leadership through variable proportional weight and improves the generalization ability of grey wolf algorithm. The specific calculation formula of variable proportional weight is as follows.

Firstly, the proportional weight calculated according to the grey wolf fitness value is as follows:

(8) $$\begin{array}{c} W_{\alpha }=\frac{F_{\alpha }}{F_{\alpha }+F_{\beta }+F_{\delta }}\\ W_{\beta }=\frac{F_{\beta }}{F_{\alpha }+F_{\beta }+F_{\delta }}\\ W_{\delta }=\frac{F_{\delta }}{F_{\alpha }+F_{\beta }+F_{\delta }}. \end{array}$$

Among them,  *F*_*α*_, *F*_*β*_, and *F*_*δ*_ represent the fitness values of grey wolves *α*, *β*, and *δ*, respectively. *W*_*α*_, *W*_*β*_, and *W*_*δ*_ represent the proportional weight of grey wolves  *α*, *β*, and *δ*, respectively. Since the above proportional weights  *W*_*α*_, *W*_*β*_, and *W*_*δ*_ are dynamically variable in each iteration process of the algorithm, the improved grey wolf algorithm can dynamically change the proportional weight according to different experimental environments, and the optimization performance and generalization are improved.

### 3.3. Neural Network Based on Improved Grey Wolf Algorithm

In the process of practical application of BP neural network, the selection of hidden layers and nodes has a great impact on the accuracy of prediction results, so it is very important to determine the number of hidden layers and nodes for the use of BP neural network. The following describes how to determine the number of hidden layers and nodes of BP neural network:

1. *Determination of Hidden Layers*. In general, 1 layer is selected for the number of hidden layers; that is, the BP neural network is a 3-layer network, which is ideal. At the same time, overfitting may also occur. Therefore, at present, selecting the number of hidden layers can achieve the ideal training effect and accuracy.
2. *Determination of the Number of Hidden Layer Nodes*. Compared with the selection of the number of hidden layers, the selection of the number of hidden layer nodes will be easier to achieve. Moreover, the determination of the number of hidden layer nodes is more important. Improper selection of the number of hidden layer nodes will make the neural network fall into local minimum, resulting in overfitting phenomenon, which will affect the prediction performance of the model. Because the improved grey wolf algorithm can effectively find the global optimal solutions of many problems and further improve the convergence speed and accuracy of the model, this study selects algorithm to optimize BP neural network. The structure diagram of BP neural network optimized by improved grey wolf algorithm is shown in Figure 4 [32].

With the continuous change in Grey wolf's position, the weight and threshold of BP neural network algorithm are constantly updated. The best position of grey wolf is the optimal solution sought by BP neural network. Through the optimization of algorithm, compared with the standard grey wolf algorithm, the effect of optimizing BP neural network is further improved. At the same time, the convergence speed and accuracy of BP neural network are further improved. The specific steps of optimizing BP neural network by algorithm are as follows:

1. The first is the selection of the structure of BP neural network itself. The most important thing is to determine the number of nodes in the network hidden layer.
2. Initialization of Basic Parameters: the grey wolf population is initialized, grey wolf position is generated, the grey wolf population size and initialization parameters *a* and *K* are calculated according to the network structure, and the maximum number of iterations is determined.
3. The fitness function of neural network and the excitation function of output node are determined.
4. The individual fitness value of grey wolf is calculated, and the optimal solution of fitness value is found.
5. Training samples and test samples for experiments are selected, and the error and its corresponding optimal solution are recorded.
6. Whether the maximum number of iterations or the set error value is met is judged, such as meeting the conditions to terminate the cycle.
7. Finally, the returned results are the position of grey wolf *α*, that is, the position of the optimal solution, the position of Grey wolf *α* in each iteration of the training process, the minimum error of the position of Grey wolf *α*, and the error of training samples and test samples.

Through the optimization of IMGWO algorithm, the feasible initial weight and the threshold of BP neural network are generated, so as to properly solve the problems of local minimum and slow convergence.

## 4. Experiments and Results

### 4.1. General Information

Sixty (60) cases of gynecological laparoscopic surgery under general anesthesia were selected in our hospital. The patient's family members before operation are informed, and signed informed consent was obtained from the patient or family members. There was no significant difference in the composition of general data such as age, body mass index, and ASA grade among the three groups (*P* > 0.05) (Table 1).

The patients were randomly divided into three groups: control group (group C), low-dose carbon dioxide group (group D1), and high-dose carbon dioxide group (group D2). Groups D1 and D2: the doses of carbon dioxide were 0.3 g and 0.6 g, respectively, diluted to 10 ml with normal saline. Group C was the control group, without carbon dioxide and 10 ml of normal saline. All patients were fasting solid food 12 hours before operation, drinking 6 hours before operation, and no preoperative drugs. After entering the room, the upper limb was opened for intravenous infusion of lactate Ringer's solution, and the Philips MP60 multifunctional monitoring system (Philips, the Netherlands) was used to monitor ECG, BP, SpO_2_, and RR. The bispectral index (BIS) module equipped with the system (Philips, the Netherlands) and aspect standard four-electrode sensor (aspect, the USA) was used to monitor BIS.

BIS monitoring method: the patient's forehead to the left temple is wiped with an alcohol cotton ball to increase the sensitivity of the sensor. No. 1 electrode of the disposable signal sensor about 5 cm is stuck above the central nasal root of the patient's forehead, a direction indication line on No. 1 electrode is made to face the nasal root, No. 2 and No. 4 electrodes are stuck above the corresponding eyebrow arch along the direction of the sensor, and finally No. 3 electrode is stuck to the Taiyang point on the same side. The sensor and power cable are connected, and self-test is started and monitored after passing the electrode impedance test.

### 4.2. Results and Analysis

The depth of sedation was assessed according to the improved OAA score. The BIS value, propofol effect chamber concentration, and hemodynamic parameters were recorded before entering the room, after pumping dexmedetomidine or normal saline and when the OAA score was stable at 4, 3, 2, and 1. Data and OAA scores were collected by the same anesthesiologist. After entering the room and before medication, the OAA score of the three groups was 5, and the BIS was greater than 94. After pumping dexmedetomidine, the OAA score of two cases and five cases in groups D1 and D2 decreased to 4 points and the BIS decreased to the range of 84 to 77. When the OAA score was stable at 4, 3, 2, and 1, the BIS values in groups D1 and D2 were significantly lower than those in group C (see Table 2). When the OAA score was 3 and 2, the BIS value of group D1 was also lower than that of group C. The value of group D2 is less than that of group D1. At OAA scores of 4, 3, and 2, group D2 was lower than group D1, and it can be seen in Table 2.

When OAA score was 4, 3, 2, and 1, the concentration of carbon dioxide effector chamber in groups D1 and D2 was lower than that in group C (*P* < 0.05) (see Table 3), and the concentration of carbon dioxide effector chamber in group D2 was lower than that in group D1 (*P* < 0.05), as shown in Figure 5.

Forearm isolation technology was prospectively studied. BIS monitoring was used to predict the recovery of consciousness after anesthesia induction. BIS was continuously monitored after intravenous injection of a single dose of propofol or thiopental, and patients were required to grasp the researcher's fingers intermittently. The results showed that although the drug concentration and duration were very inconsistent, it was consistent that consciousness began to recover when BIS increased more than 60; the BIS value below 65 indicates that the possibility of consciousness recovery within 50 seconds is not N5%. No patient who responded to the command can recall this episode. This study supports that BIS value is a good indicator to judge whether the patient's consciousness is restored. The incidence of respiratory depression and hypotension in group C was significantly higher than that in groups D1 and D2. Compared with group C, the incidence of bradycardia in groups D1 and D2 is higher, and the incidence of bradycardia in group D2 is higher than that in group D1 (see Figure 6).

## 5. Conclusion

Anesthesiology is developing rapidly. The diversification of anesthetics, the renewal of anesthesia equipment, and the improvement of operation methods have put forward new challenges and requirements for anesthesiologists. The rationalization, refinement, and individualization of drug use have also become the common goal of anesthesiologists. Good anesthesia has several elements: sufficient sedation, reasonable analgesia, and satisfactory muscle relaxation. Among them, adequate sedation is an important premise to ensure the comfort and safety of patients and the smooth completion of surgery. Patients have a higher and higher demand for “painless,” not only in routine surgery but also in some interventional radiotherapy and endoscopy. Good sedation and analgesia have also become an urgent demand for patients.

The traditional evaluation method cannot meet the needs of clinical work. Studies have shown that there is no direct correlation between changes in consciousness and hemodynamic parameters such as heart rate and blood pressure. In particular, in the case of combined medication, the changes in hemodynamics cannot accurately reflect the sedation degree of drugs. At present, many evaluation methods of sedation depth are widely used in clinics, and alert sedation score (OAA/s) is one of the commonly used methods in clinic. As a commonly used sedation depth monitoring index in clinics, the results of BIS are very useful for the judgment of sedation depth. However, it cannot be called an ideal sedation depth detection index.

This study also has some limitations. The sample size is relatively small. We are patients who choose gynecological laparoscopic surgery under certain conditions, which can eliminate the tension and anxiety caused by patients without ideological preparation. In this study, the method of single administration of carbon dioxide is adopted, so we can only see the influence of carbon dioxide on BIS value after single administration. Then, when the constant load dose of carbon dioxide is given and continuously pumped, we have not done research.

## Figures and Tables

**Figure 1:** Schematic diagram of EEG signal and bispectral index.

**Figure 2:** Representation of basic EEG monitoring [19].

**Figure 3:** Grey wolf algorithm flow chart.

**Figure 4:** Improved grey wolf algorithm to optimize BP neural network structure diagram [29].

**Figure 5:** Propofol effect chamber concentration corresponding to different OAA scores in group A.

**Figure 6:** Comparison of adverse events of respiration and circulation among the three groups.

**Table 1:** Comparison of general conditions and indexes of three groups of patients.

Group	Age	Body mass index	Hierarchical structure
C	49 ± 9	23 ± 3	9/11
D1	52 ± 7	23 ± 4	12/8
D2	50 ± 6	22 ± 3	10/10

**Table 2:** Comparison of BIS values and OAA scores among the three groups.

	OAA score					
	T0	T1	1	2	3	4
C	97 ± 1	96 ± 3	82 ± 4	65 ± 3	59 ± 4	46 ± 5
D1	96 ± 1	93 ± 3	80 ± 4	59 ± 6	54 ± 4	42 ± 3
D2	97 ± 1	91 ± 3	73 ± 4	53 ± 3	48 ± 4	39 ± 3

**Table 3:** Comparison of BIS values and OAA scores among the three groups.

	4	3	2	1
C	1.11 ± 0.38	1.52 ± 0.37	1.70 ± 0.25	1.88 ± 0.06
D1	0.82 ± 0.26	1.14 ± 0.19	1.33 ± 0.11	1.62 ± 0.08
D2	0.25 ± 0.11	0.45 ± 0.15	0.66 ± 0.07	0.73 ± 0.03

## Data Availability

The datasets used during this study are available from the corresponding author on reasonable request.
